This article has been retracted.

# Hypoxia-Inducible MiR-210 Is an Independent Prognostic Factor and Contributes to Metastasis in Colorectal Cancer

**DOI:** 10.1371/journal.pone.0090952

**Published:** 2014-03-14

**Authors:** Ailin Qu, Lutao Du, Yongmei Yang, Hui Liu, Juan Li, Lili Wang, Yimin Liu, Zhaogang Dong, Xin Zhang, Xiumei Jiang, Haiyan Wang, Zewu Li, Guixi Zheng, Chuanxin Wang

**Affiliations:** Department of Clinical Laboratory, Qilu Hospital, Shandong University, Jinan, Shandong Province, China; IRCCS-Policlinico San Donato, Italy

## Abstract

MicroRNA-210 (miR-210), the master hypoxamir, plays pleiotropic roles in certain cancers; however, its role in the development of human colorectal cancer remains unclear. Herein, we report that miR-210 is frequently up-regulated in colorectal cancer tissues, with high miR-210 expression significantly correlating with large tumor size, lymph node metastasis, advanced clinical stage and poor prognosis. Functionally, miR-210 overexpression promotes the migration and invasion of colorectal cancer cells. Furthermore, miR-210 can be induced by hypoxia and mediates the hypoxia-induced metastasis of colorectal cancer cells. In addition, vacuole membrane protein 1 (VMP1) is identified as the direct and functional target of miR-210. Thus, miR-210 is a useful biomarker for hypoxic tumor cells and a prognostic factor that plays an essential role in colorectal cancer metastasis.

## Introduction

Colorectal cancer (CRC) remains the third most common malignancy worldwide and accounts for the fifth leading cause of cancer-related death in China [1]. Although recent improvements in diagnostic techniques and clinical management have increased the early detection of CRC and decreased the mortality rate, approximately 25% of CRC patients present with stage IV disease [1]. Moreover, patients with advanced disease frequently develop recurrent disease following extended radical resections, consequently showing extremely poor survival rates due to metastasis [2], and the 5-year postsurgical survival rate falls from 90% to 10% or even less after metastasis has occurred. A growing number of studies have demonstrated that both tumor cells and micro-environmental factors orchestrate the critical events that lead to metastasis [3], thereby emphasizing the need to further understand the tumor microenvironment and molecular mechanisms involved in tumor metastasis.

Hypoxia, or low oxygen tension, is a common feature of solid tumor microenvironment. Hypoxic tumors tend to be more aggressive, more likely to metastasize, more resistant to conventional therapies, and are associated with a poor prognosis [4]–[6]. The gene encoding HIF1 (hypoxia-inducible factor-1), which is composed of the HIF1α and HIF1β subunits, is perhaps the most studied gene that plays an essential role in the response to hypoxia [7]. HIF1α is stable under hypoxic conditions, with its expression rapidly decreasing under normoxic conditions, whereas HIF1β is constitutively expressed under both conditions [8]. Evidence is accumulating regarding the significance of HIF1α expression in various solid tumors [9]–[11], and increased HIF1α expression has recently been reported to contribute to colorectal cancer metastasis [12], [13].

MicroRNAs (miRNAs, miRs) are a novel class of endogenous, small, non-coding RNA oligonucleotides that regulate gene expression by targeting the 3′ untranslated region (3′-UTR) of the corresponding mRNA [14], [15]. Dysregulation of miRNAs is a well-known key process in the pathogenesis of many cancers and can occur at any point, from initiation to metastasis. There is a functional link between hypoxia and microRNA dysregulation in cancer. For instance, Chen H has reported that miR-103/107 was increased in the presence of hypoxia and could contribute to hypoxia-stimulated metastasis in CRC [16]. Many microRNAs, such as miR-21, 93, 103, 107, 192, 195, 210, and 213, can be induced and markedly up-regulated by HIF1α in cancer cells under hypoxic conditions [17], [18]. Among the miRNAs induced by HIF1α, miRNA-210 is the most prominent and consistently up-regulated miRNA during the hypoxic response in different types of tumor cells and normal cells [19], [20]. Recently, Ying et al. showed that hypoxia-induced miR-210 could enhance the migration and invasion of hepatocellular carcinoma (HCC) [21], and Redova and colleagues found that the downregulation of miR-210 inhibited the migratory and invasive potential of renal cell carcinoma (RCC) [22], Rothé reported similar results in breast cancer [23]. Most studies have shown that miR-210 may act as an oncogenic miRNA and is associated with a poor prognosis in some human epithelial cancers [21], [24]–[26]. However, a few studies have indicated that miR-210 expression is lost during tumorigenesis and that the miRNA exerts a tumor-suppressor effect on human epithelial ovarian and esophageal squamous cell carcinoma [27], [28]. These data indicate that miR-210 may play crucial roles during tumorigenesis and cancer progression and may exert various effects on different cancers. Although it has been reported that miR-210 is expressed and greatly up-regulated in response to hypoxia in CRC cell lines (HCT-116 and HT-29), the function of miR-210 in colorectal cancer has not been elucidated to date, and its role in colorectal cancer progression remains unclear.

In the current study, we focused on miR-210, the hypoxia-induced miRNA, and examined its expression in human CRC tissues, analyzed its correlation with clinicopathological characteristics and prognosis, and then uncovered the role of miR-210 in hypoxia-induced metastasis during colorectal cancer progression.

## Materials and Methods

### Patients and tissue samples

Tissue samples, including tumor tissues and adjacent non-cancerous tissues, were obtained from 193 CRC patients at the time of surgery at the Department of General Surgery, Qilu Hospital of Shandong University, Jinan, China, from June 2003 to February 2008. None of the patients had ever received any chemotherapy, radiotherapy, or surgery. All the tissues were immediately placed in liquid nitrogen and frozen at −80°C until RNA extraction. This study was approved by the Ethical Committee of Qilu Hospital, Shandong University, and written informed consent was obtained from each patient.

The clinicopathological data, including sex, age, tumor location, tumor stage, tumor size, local invasion, histological differentiation and lymph node metastasis were collected retrospectively. The duration of follow-up was calculated from the date of surgery to death or last follow-up, and we completed the follow-up in April 2012. The patients were excluded from analysis of clinicopathological characteristics and prognosis if they had incomplete medical records or inadequate follow-up.

### Cell culture

CRC cell lines (HT-29, SW480, and SW620) and HEK (human embryonic kidney) 293T cell line were purchased from the Type Culture Collection of the Chinese Academy of Sciences (Shanghai, China), and the HCT116 cell line was purchased from Shanghai Institute of Biochemistry and Cell Biology (China). All the cell lines were cultured in Dulbecco's modified Eagle's medium (DMEM; Hyaline, Logan, UT) containing 10% fetal bovine serum (FBS; Gibco, Carlsbad, CA) at 37°C in a 5% CO_2_ incubator. To induce hypoxia, the cells were exposed to a steady flow of a low-oxygen gas mixture (1% O_2_, 5% CO_2_, and 94% N_2_) in a humidified incubation chamber (MiniGalaxy, RSBiotech, Irvine, Scotland).

### RNA isolation, cDNA synthesis, and quantitative real-time polymerase chain reaction (qRT-PCR)

Total RNA was extracted using TRIzol reagent (Invitrogen, Carlsbad, CA) according to the manufacturer's protocol. All of the manipulations of the RNA were carried out under RNase-free conditions. RNA concentration was measured using a BioPhotometer plus (Eppendorf, Hamburg, Germany) at 260 nm, and the isolated RNA was stored at −80°C until use. For the analysis of HIF1α and VMP1mRNA expression, total RNA (1 μg) was reverse transcribed into cDNA using the SuperScript kit (Toyobo, Osaka, Japan), and qRT-PCR analyses were performed using SYBR Green (Toyobo, Osaka, Japan) and an ABI PRISM 7500 Sequence Detection System (Applied Biosystems, Foster City, CA). The fold changes in HIF1α and VMP1 mRNA expression were quantified using the 2^−ΔΔCT^ relative quantification method with β-actin as a housekeeping control. The primers for β-actin (forward primer: 5′-TGGAGTCCTGTGGCATCCACGAAA-3′, reverse primer: 5′-TGTAACGCAACTAAGTCATAGTCCG-3′), HIF-1α (forward primer: 5′-ATCGCGGGGACCGATT-3′, reverse primer: 5′-CGACGTTCAGAACTTATCTTTTTCTT-3′) and VMP1 (forward primer: 5′-GAGATGCTGGAACATGCAGA-3′, reverse primer: 5′-TTGCTCCACTATGTGCTTGC-3′) were purchased from BioSune, Shanghai, China. For miRNA expression, cDNA was synthesized using gene-specific primers (Ribobio, Guangzhou, China) and the M-MLV RT kit (Invitrogen, Carlsbad, CA, USA) in a 20-μl reaction volume. The RT reaction reagents contained 1 μg RNA template, 1 μl 10 mM dNTP mix, 2 μl 0.1 M DTT, 4 μl 5× first-strand buffer, and 1 μL 40 U/μl RNase inhibitor. The volume was adjusted with RNA-free H_2_O. The reverse-transcription reaction was performed in triplicate to remove any outliers. MiRNA expression was assessed using qRT-PCR and an ABI PRISM 7500 Sequence Detection System (Applied Biosystems, Foster City, CA). The fold changes in miRNA expression were determined using the 2^−ΔΔCT^ method; the expression was normalized to the U6 small nuclear RNA (U6) expression level. In addition, the relative expression of miRNA, HIF1α and VMP1 in HT-29 cells severed as calibrator in each run and was set at the value of 1.

### Transfection with miRNA/plasmid

CRC cells were plated at a density of 5×10^4^ cells/well in 24-well plates or at 1.5×10^5^ cells/well in 6-well plates and were cultured approximately 24 h before transfection. After the cells reached 50% confluence, transient transfection of miRNA mimics/inhibitor (RiboBio, Guangzhou, China) and/or plasmid were carried out using Lipofectamine 2000 (Invitrogen, Carlsbad, CA, USA) following the manufacturer's instructions. For each experiment, the transfection efficiencies were evaluated by qRT-PCR at 24 h after transfection.

### Migration and invasion assays in vitro

Transwell chambers (diameter of 6.5 mm, pore size of 8 μm) (Corning, NY, USA) coated with or without Matrigel (BD Biosciences, Franklin Lakes, NJ, USA) were used to perform the migration and invasion assays. At 24 h post-transfection, the HT-29 (5×10^4^ cells) or SW480 (1×10^5^ cells) cells were resuspended in a medium containing 1% FBS and placed in the top chamber of each insert. An aliquot of medium containing 10% FBS (500 μl) was added to the lower chambers. After incubation for 24 h at 37°C, the cells adhering to the lower membrane were stained with 0.1% crystal violet, imaged (200×), and counted using an IX81 inverted microscope (Olympus, Tokyo, Japan).

### Luciferase assay

Luciferase reporter assay was carried out using the pmiR-REPORTTM vectors (RiboBio, Guangzhou, China) containing wild type (WT)-VMP1 3′-UTR sequences or mutant (MUT)-VMP1 3′-UTR sequences. HEK293T cells were transiently cotransfected with miR-210 mimics/miR-negative control and WT-VMP1 3′-UTR vector/MUT VMP1 3′-UTR vector. Luciferase activities were measured using the Dual-Luciferase assay kit (Promega, Madison, WI) according to manufacturer's instructions 48 h after transfection.

### Western blot

Total protein of cultured cells was extracted by RIPA buffer containing PMSF. BCA protein assay kit (Beyotime, Haimen, China) was used to determine the concentration. Proteins was separated via SDS-PAGE and transferred onto PVDF membranes. After blocking, the membrane was incubated with mouse anti-VMP1 polyclonal antibody (Abcam, Southampton, UK) or anti-β-actin mouse monoclonal antibody (Santa Cruz Biotechnology, Santa Cruz, CA, USA), followed by incubation with HRP-conjugated secondary antibodies (Santa Cruz Biotechnology, Santa Cruz, CA, USA). Signals were determined by a chemiluminescence detection kit (Amersham Pharmacia Biotech, Piscataway, NJ).

### Statistical analysis

The SPSS (Statistical Package for the Social Sciences) software package, version 18.0 (Chicago, IL, USA), was used to analyze all the data. We first used the Kolmogorov-Smirnov test to determine the distribution of the data in each group. The data are presented as the mean ± standard deviation (SD) or median (interquartile range) when the values were normally or abnormally distributed, respectively. Statistical differences between the groups were tested using the Mann-Whitney *U*-test, Student's *t*-test, or a Kruskal-Wallis test, as appropriate. The correlation between miR-210 and HIF1α (or VMP1) was determined by Pearson's correlation analysis. The Kaplan-Meier method was used to estimate survival, and the survival differences between the subgroups were examined using the log-rank test. A Cox regression model (Proportional hazard model) was applied for the univariate analysis and multivariate analysis of prognostic factors. Differences were considered statistically significant only when *P*<0.05.

## Results

### MiR-210 is frequently up-regulated in colorectal cancer tissues and involved in CRC development

The expression levels of miR-210 in 193 pairs of human CRC tissues and corresponding non-cancerous tissues were examined using qRT-PCR. In order to ensure that the reference gene U6 does not change between tumor tissues and corresponding non-cancerous tissues, we calculated the mean Ct values as 2^-ct^. The level of U6 did not show any significant differences between tumor and corresponding non-cancerous samples (2^-CtTumor^/2^-CtNon-cancerous^ = 0.93; *P* = 0.34) (Figure S1). The results indicated that miR-210 expression in the CRC tissues was significantly up-regulated in comparison to that in the adjacent normal tissues (*P*<0.001, Fig. 1A). In addition, 58% (111 of 193) of the samples displayed more than 2-fold upregulation of miR-210 compared to the non-cancerous tissue samples, implying that the overexpression of miR-210 is a common event in CRC. In a controlled experiment, we also found miR-21, another overexpressed miR in CRC [29], was significantly up-regulated in CRC tissues compared with adjacent non-tumor tissues (*P*<0.001, Figure S2), confirming the feasibility and reliability of our method. Moreover, HIF1α expression in CRC tissues was up-regulated (*P*<0.001; Figure 1D) and positively correlated with miR-210 expression in CRC tissues (r = 0.402, *P*<0.01; Fig. 1E).

**Figure 1:** MiR-210 expression is increased in CRC tissues and associated with a poor prognosis. (A) MiR-210 expression was tested using qRT-PCR in 193 pairs of human CRC tissues (CRC) and adjacent non-tumorous tissues (NT), and its expression was normalized to the level of U6 small nuclear RNA (U6) expression in each sample. (B) Fold changes in miR-210 expression in each paired sample. The data are represented as a log_2_-fold change (cancer/normal), which was defined as >1 (overexpression) and <−1 (underexpression); the remaining fold changes were defined as unchanged. (C) The overexpression of miR-210 was found in 58% (111 of 193) of the CRC tissues compared to the adjacent non-tumorous tissues. (D) HIF1α mRNA expression was detected in CRC tissues (CRC) and adjacent non-tumorous tissues (NT), and its expression was normalized to the level of β-actin expression in each sample. (E) The correlation between miR-210 expression and HIF1α mRNA levels in CRC tissues was analyzed using Pearson's correlation analysis. (F) Kaplan-Meier overall survival curves according to the level of miR-210 expression. The patients with high miR-210 expression had a significantly poorer 5-year overall survival rate than those with low miR-210 expression (*P*<0.001). The median miR-210 expression level in the tumor samples was chosen as the cut-off point.

We further summarized the association of miR-210 expression levels with various clinicopathological characteristics in CRC tissues and found that miR-210 expression was significantly correlated with large tumor size (*P* = 0.014), local invasion (*P* = 0.047), positive regional lymph node metastasis (*P* = 0.001), and TNM stage (*P* = 0.005). However, there were no significant associations between miR-210 expression and the patient's gender, age, tumor location, or histology grade (all *P*>0.05). The detailed results of the statistical tests between miR-210 expression and the clinicopathological characteristics are listed in Table 1.

**Table 1:** MiR-210 expression and clinicaopathological feature in CRC patients.

Clinicopathological feature	NO. of cases	miR-210 expression	*P*
Age			0.209
<59	57	39.005 (19.749–84.122)	
≥59	59	54.629 (28.670–86.528)	
Gender			0.185
Male	64	39.420 (20.501–78.030)	
Female	52	50.693 (28.670–93.932)	
Tumor location			0.152
Colon	54	48.128 (29.406–110.806)	
Rectum	62	45.206 (19.412–70.744)	
Tumor size (cm)			0.014
<4.7	60	37.152 (23.305–68.094)	
≥4.7	56	57.727 (28.592–107.616)	
Histology grade			0.528
Poor	15	39.005 (28.670–69.186)	
Moderate	83	46.057 (19.086–77.122)	
Well	11	57.536 (38.092–91.122)	
Local invasion			0.047
T1–T2	19	38.092 (18.048–47.377)	
T3	37	45.903 (18.261–89.718)	
T4	58	52.915 (29.858–105.595)	
Lymph node metastasis			0.001
NO	53	39.004 (18.528–56.640)	
YES	63	57.918 (29.807–121.669)	
TNM stage			0.005
I	17	40.092 (18.528–51.877)	
II	36	37.418 (17.784–59.038)	
III	57	57.536 (28.438–117.372)	
IV	6	122.584(30.557–166.426)	

### MiR-210 is an independent prognostic marker for the overall survival of CRC patients

A total of 50 patients died during the follow-up period, and the cumulative 5-year overall survival rate was 56.9%. Using the median of the miR-210 expression levels as a cutoff, we divided the 116 CRC patients into two groups: a high miR-210 expression group and a low miR-210 expression group. We then used the Kaplan-Meier survival curve analysis to assess the prognostic value of miR-210 in colorectal cancer. The results showed that the patients with high miR-210 expression had a significantly poorer prognosis than those with low miR-210 expression (*P*<0.001, Fig. 1F). To evaluate whether miR-210 expression was an independent indicator of overall survival for CRC patients, we first applied a univariate Cox proportional hazards regression model to estimate the individual hazard ratio for all of the clinicopathological parameters. The results showed that overall survival was significantly related to the miR-210 expression level (RR = 2.621; 95% CI, 1.457–4.712; *P* = 0.001) and other four parameters (tumor size, local invasion, regional lymph node metastasis, and TNM stage; all *P*<0.05). In the multivariate analysis, the Cox proportional hazards model involving the five significant prognostic factors identified miR-210 expression as an independent prognostic factor for patients with CRC (*P* = 0.008). The statistical values of miR-210 expression and the other clinicopathological parameters derived from the Cox proportional hazards regression model are listed in Table 2.

**Table 2:** Univariate and multivariate analysis of overall survival in colorectal cancer patients.

Clinicopathological feature	Univariate analysis			Multivariate analysis		
	HR	95%CI	*P* value	RR	95%CI	*P* value
**Age**	0.822	0.471–1.435	0.491			
**Gender**	1.026	0.587–1.794	0.928			
**Tumor location**	0.767	0.440–1.336	0.348			
**Size**	1.759	1.002–3.085	0.049	1.756	0.961–3.209	0.067
**Differentiation**	0.884	0.506–1.545	0.665			
**Local invasion**	0.885	0.789–0.991	0.035	1.106	0.965–1.267	0.146
**Lymph node metastasis**	3.653	1.936–6.896	<0.001	0.451	0.131–1.557	0.208
**TNM stage**	3.200	1.997–5.130	<0.001	5.613	2.365–13.319	<0.001
**miR**–**210 expression**	2.621	1.457–4.712	0.001	2.131	1.130–4.019	0.019

### MiR-210 is expressed in CRC cell lines and is induced by hypoxia in CRC cells

We examined the expression level of miR-210 in a panel of CRC cell lines, including HCT-116, HT-29, SW620 and SW480. The results showed that the level of miR-210 was highest in HT-29 cells compared with the other three cell lines, and its level was lowest in SW480 cells (Fig. 2A). Based on this expression pattern, we therefore chose HT-29 and SW480 for the following studies. As presented in Figure 2D and 2E, we found that the miR-210 levels increased in response to hypoxia in these cells. Moreover, the expression of miR-210 greatly increased with prolonged exposure to hypoxia, indicating that miR-210 was indeed induced by hypoxia in CRC cell lines.

**Figure 2:** MiR-210 is induced by hypoxia in CRC cell lines. (A) MiR-210 expression in CRC cell lines. (B, C) HIF1α mRNA expression in HT-29 (B) and SW480 (C) cells under hypoxic conditions. (D, E) MiR-210 expression in HT-29 (D) and SW480 (E) cells under hypoxic conditions. The data are presented as the mean of three measurements, and the error bars represent the SD of the mean. *P<0.05.

### MiR-210 promotes CRC cell migration and invasion and mediates the hypoxia-induced migration and invasion of CRC cells

To measure the biological properties of miR-210 in CRC cells, we transiently modulated the miR-210 expression level by transfection with miR-210 mimics or inhibitor. As shown in Figure 3, the transfection efficiency was very high in the HT-29 and SW480 cell lines. Transwell experiments with or without Matrigel were performed to test the effect of miR-210 on CRC cell migration and invasion, and we found that the upregulation of miR-210 by the miR-210 mimics enhanced the migration and invasion ability of CRC cells (Fig. 4A, 4C). In accordance with these results, transfection with the miR-210 inhibitor led to a significant decrease in the migration and invasion ability of CRC cells compared to the cells transfected with the miR negative control (Fig. 4B, 4D). Taken together, our observations indicate that miR-210 could promote the migration and invasion ability of CRC cells.

**Figure 3:** Transfection efficiency assays. (A, C) MiR-210 expression in HT-29 (A) and SW480 (C) cells was significantly increased after transfection with the miR-210 mimics. (B, D) MiR-210 expression in HT-29 (A) and SW480 (C) cells was greatly decreased after transfection with the miR-210 inhibitor. The data are presented as the mean of three measurements, and the error bars represent the SD of the mean. *P<0.05 compared to the corresponding negative control.

**Figure 4:** MiR-210 promotes the migration and invasion ability of CRC cells. (A, B) Transwell migration assays of HT-29 and SW480 cells were performed after transfection with the miR-210 mimics (A) or inhibitor (B). (C, D) Transwell invasion assays of HT-29 and SW480 cells were performed after transfection with the miR-210 mimics (C) or inhibitor (D). In all panels, the results are representative of at least three independent experiments. NC, negative control.

Because we demonstrated miR-210 could increase the migration and invasion potential of CRC cells, we hypothesized that miR-210 could also mediate the hypoxia-induced migration and invasion of CRC cells. To confirm this hypothesis, we performed transwell assays to examine the migration and invasion potential of CRC cells under hypoxic conditions and found that the migration and invasion ability of these CRC cells were significantly increased compared to cells under normoxic conditions. Moreover, transfection with the miR-210 inhibitor dramatically diminished the migration and invasion ability of the hypoxic CRC cells, whereas transfection with the miR-210 mimics further enhanced the migration and invasion ability of the CRC cells (Fig. 5). The above results demonstrate that miR-210 plays an important role in the hypoxia-induced migration and invasion of CRC cells.

**Figure 5:** MiR-210 mediates the hypoxia-induced migration and invasion ability of CRC cells. (A, B) Transwell migration and invasion assays of HT-29 and SW480 cells were performed after transfection with the miR-210 mimics or the negative control (NC) under normoxic or hypoxic conditions. (C, D) Transwell migration and invasion assays of HT-29 and SW480 cells were performed after transfection with the miR-210 inhibitor or the negative control under normoxic or hypoxic conditions. In all panels, the results are representative of at least three independent experiments.

### VMP1 is a direct target of miR-210

TargetScan identifies that 3′-UTR of VMP1 contains predicted binding site for miR-210 (Fig. 6A). Luciferase activity assay showed that miR-210 significantly inhibited the luciferase activity of the WT 3′-UTR but not the Mut 3′-UTR of VMP1 in HEK293T cells (Fig. 6B). Furthermore, overexpression of miR-210 significantly inhibited VMP1 mRNA and protein levels in HT-29 and SW480 cells (Fig. 6C, 6D) and VMP1 level was inversely correlated with miR-210 expression in primary CRC tissues (r = −0.318, *P*<0.01; Fig. 6E). These data strongly suggest that miR-210 negatively regulates VMP1 expression by directly targeting its 3′-UTR sequences.

**Figure 6:** MiR-210 suppresses VMP1 expression by directly binding to its 3′-UTR. (A) The putative miR-210 binding sequences in VMP1 3′-UTR. (B) Luciferase activity assay was performed for the HEK293T cells cotransfected with pmiR-REPORT™ vectors containing WT-VMP1 3′-UTR or MUT-VMP1 3′-UTR sequences and miR-210 mimics. Data are presented as normalized fold change in luciferase activity. (C, D) VMP1 mRNA and protein were determined in HT-29 cells and SW480 cells transfected with miR-210 mimics or miR-negative control by qRT-PCR and Western blot, respectively. (E) Inverse correlation between miR-210 expression and VMP1 mRNA levels in CRC tissues was analyzed using Pearson's correlation analysis.

### Overexpression of VMP1 partially reverses the migration and invasion of CRC cells induced by miR-210

To determine whether VMP1 is involved in the miR-210 induced metastasis of CRC cells, we performed rescue assays. As shown in Figure 7, miR-210 mimics could augment the metastatic ability of CRC cells and decreased metastatic potential was observed in VMP1-overexpressing cells compared with control cells. Furthermore, concomitant overexpression of miR-210 and VMP1 could partially abrogate miR-210-induced metastatic potential in CRC cells. These results demonstrate that miR-210 can promote CRC cell migration and invasion by targeting VMP1.

**Figure 7:** Overexpression of VMP1 partially reverses the migration and invasion of CRC cells induced by miR-210. (A, B) Transwell migration and invasion assays were performed in VMP1-overexpressing HT-29 cells cotransfected with miR-210 mimics or negative control. (C, D) Transwell migration and invasion assays were performed in VMP1-overexpressing SW480 cells cotransfected with miR-210 mimics or negative control. In all panels, the results are representative of at least three independent experiments.

## Discussion

Hypoxia is a prevalent characteristic feature of most solid tumors, and the robust hypoxia-induced miRNA, miR-210 is currently regarded as the “master miRNA” of the hypoxia response [15]. Accordingly, it is important to explore the potential roles of miR-210 in solid tumor progression, as this miRNA has been proven to play a key role in the development of cancer under hypoxic conditions [21], [30]. Our results provide the first evidence that miR-210 is overexpressed in CRC tissues and functions as a key factor in the progression of CRC.

The dysregulated expression of miR-210 has been irrefutably demonstrated in different human malignancies. Cai et al. showed that miR-210 expression was significantly higher in pediatric osteosarcoma patients and was significantly associated with aggressive clinicopathological features and a poor prognosis [31]. However, Tsuchiya [32] reported that miR-210 expression was markedly downregulated in patients with poorly differentiated esophageal squamous cell carcinoma. In contrast, Greither et al. [33] reported that there were no statistically significant correlations between miR-210 expression and any aggressive clinicopathological features in soft-tissue sarcoma. These discordant findings may be explained by the various roles that miR-210 might play in the pathogenesis of different cancers. Here, we detected a marked upregulation of miR-210 expression in CRC tissues, and miR-210 overexpression was significantly correlated with aggressive clinicopathological features, such as a large tumor size, positive regional lymph node metastasis, local tumor invasion, and an advanced clinical stage. We also found that miR-210 level was positively correlated with HIF1α expression that was related to metastasis and unfavorable prognosis of CRC [12], [13]. These findings indicated that miR-210 may play important roles in the development of the progressive phenotype of CRC.

With regard to survival, univariate and multivariate analyses were performed to explore the potential prognostic value of miR-210 in CRC. The results of the univariate analysis showed that patients with higher miR-210 levels had a poorer prognosis than those with a lower miR-210 level. Furthermore, the results of the multivariate analysis of the Cox proportional hazards regression model showed that miR-210 was an independent prognostic factor for overall patient survival after surgery. These results are in agreement with the studies reported by Camps et al. in breast cancer [34] and Gee et al. in head and neck cancer [35]. Together with our results, these findings indicate that miR-210 could be a promising prognostic marker to identify patients with a poor prognosis.

The functional exploration of miR-210 indicated that miR-210 plays key roles in many cellular processes involved in physiological and malignant conditions. MiR-210 may be involved in erythropoiesis and can also promote adipogenesis [36], [37]. As the most consistently and robustly up-regulated miRNA under hypoxic conditions, miR-210 regulates many aspects of hypoxia pathways, such as the angiogenic response of endothelial cells to hypoxia [38]. Consistent results have shown that the up-regulated expression of miR-210 is involved in the hypoxia/VEGF signaling pathway in breast cancer [34]. In epithelial ovarian cancer, however, miR-210 is often deleted and may inhibit cell cycle progression [27].

In the present study, we found that the overexpression of miR-210 markedly promoted the migration and invasion of CRC cells. Our data imply that miR-210 acts as an oncogenic miRNA in human colorectal cancer to promote metastasis, which is consistent with the findings of earlier studies [21]-[23]. We also confirmed previous findings that showed that miR-210 was up-regulated in CRC cells in response to hypoxia and that miR-210 was induced in a time-dependent manner. These results indicate that miR-210 is also a hypoxic marker in CRC patients, as it is in other cancers, such as head and neck cancer [35]. Furthermore, we found that miR-210 mediated the hypoxia-induced migration and invasion of CRC cells. Thus, in addition to its roles in the adaption of tumor cells to low-oxygen stress and as a marker for tumor hypoxia, we suggest that elevated levels of miR-210 may have biological functions associated with the malignancy and metastasis of tumors, potentially explaining why miR-210 is associated with a poor prognosis in cancer patients. Further investigation revealed that VMP1 was the functional down-stream target of miR-210 in CRC. VMP1 is a transmembrane protein localized to intracellular vacuoles that was originally described as a protein associated with acute pancreatitis [39]. In kidney cancer metastases and metastatic breast cancer cell lines, VMP1 is reduced [40]. And in HCC, VMP1 is identified as a downstream target of miR-210 and the reduced VMP1 correlates with tumor metastases [21]. In accordance with these studies, we found that VMP1 is also reduced in CRC samples and acts to suppress tumor metastatic potential. These results indicated that miR-210 directly downregulated the expression of VMP1 and consequently inhibited metastasis of CRC cells. However, overexpression of VMP1 partially reversed the migration and invasion of CRC cells induced by miR-210. This could be due to the fact that one miRNA normally targets a great amount of mRNAs whereas one mRNA can be potentially regulated by multiple miRNAs [41]. Further studies are needed to reveal the network between miR-210 and other targeted genes, which will provide a more detailed insight to understand the molecular mechanism of the function of miR-210.

## Conclusions

We found that miR-210 upregulation was correlated with aggressive tumor progression in CRC and that it could be used in the prognostic screening of patients with this malignancy. Moreover, we found that the “master” microRNA in hypoxia control, miR-210, is frequently up-regulated in CRC cells and is involved in hypoxia-induced CRC metastasis. These results add to the accumulating evidence that miR-210 plays a critical role in promoting cancer development and may assist in the development of new therapeutic regimens against hypoxic tumors.

## Supporting Information

Figure S1 **Evaluation of the reference gene U6 variations between tumor tissues and corresponding non-cancerous tissues.** There are no differences in U6 expression between the two groups (*P* = 0.34).
(TIF)

Figure S2 **MiR-21 relative expression level in CRC tissues (CRC) and adjacent non-tumorous tissues (NT).** The miR-21 level was significantly higher in CRC tissues than in adjacent non-tumorous tissues, and its expression was normalized to the level of U6 small nuclear RNA (U6) expression in each sample.
(TIF)
